The article "Identification of an m6A RNA Methylation Regulator Risk Score Model for Prediction of Clinical Prognosis in Astrocytoma" was retracted in 2023. Reasons: signs of a paper mill; compromised peer review; unreliable results or conclusions.

# Identification of an m6A RNA Methylation Regulator Risk Score Model for Prediction of Clinical Prognosis in Astrocytoma

**DOI:** 10.1155/2022/7168929

**Published:** 2022-01-10

**Authors:** Fangzhou Guo, Teng Deng, Liu Shi, Pinghua Wu, Jun Yan, Guoyuan Ling, Hainan Chen, Qianrong Huang, Junbo Mu, Ligen Mo

**Affiliations:** Department of Neurosurgery, Affiliated Tumor Hospital of Guangxi Medical University, Nanning, Guangxi, China

## Abstract

Astrocytoma (AS) is the most ubiquitous primary malignancy of the central nervous system (CNS). The vital involvement of the N6-methyladenosine (m6A) RNA modification in the growth of multiple human tumors is known. This study entailed probing m6A regulators with AS prognosis to construct a risk prediction model (RS) for potential clinical use. A total of 579 AS patients' (of the Chinese Glioma Genome Atlas,CGGA) data and the expression of 12 published m6A-related genes were included in this study. Cox and selection operator (LASSO) regression analyses for independent prognostic factors and multifactor Cox analysis established an R.S. model to predict the AS patient prognosis. This was subject to verification employing 331 samples from the TCGA data set followed by gene ontology and pathway enrichment study with gene set enrichment analysis (GSEA). The R.S. constructed with three m6A genes inclusive of WTAP, RBM15, and YTHDF2 emerged as independent prognostic factors in AS patients with vital involvement in the advancement and development of the malignancy. In a nutshell, this work reported an m6A-related gene risk model to predict the prognosis of AS patients to pave the way for discerning diagnostic and prognostic biomarkers. Further corroboration employing relevant wet-lab assays of this model is warranted.

## 1. Introduction

Astrocytoma (AS) is the most ubiquitous intracranial malignancy, accounting for 40-50% of primary CNS tumors. AS is categorized by the WHO (World Health Organization) as pilocytic astrocytoma, diffuse astrocytoma, anaplastic astrocytoma, and glioblastoma (grade-I, grade-II, grade-III, and grade-IV, respectively) [1, 2]. Most tumors document a higher recurrence rate post-esection with the occurrence of a higher grade and more aggressive tumor type in the event of relapse. Notwithstanding the extensive use of comprehensive treatment approaches inclusive of surgical resection, radiotherapy, and chemotherapy, the 5-year survival rate of highly aggressive AS is still less than 20%. Another roadblock is the high disability rate after surgery that seriously impacts the patients' quality of life [3]. In comparison, prognosis prediction and treatment guidance employ traditional clinical risk factors, including tumor grade, preoperative imaging, and IDH gene silencing status. Useful molecular indicators as possible treatment targets have yet to be discovered [4, 5].

The article "Identification of an m6A RNA Methylation Regulator Risk Score Model for Prediction of Clinical Prognosis in Astrocytoma" was retracted in 2023. Reasons: signs of a paper mill; compromised peer review; unreliable results or conclusions.

The m6A methylation of RNA is modified at the N6-position of the adenine base via methyl transferase catalysis. Currently, this is the most ubiquitous mRNA modification scrutinized in eukaryotic cells and is receiving the center stage in current research [6–8]. The genetic information carried on DNA is first transcribed into mRNA and then further translated into functional proteins. m6A is vitally involved in controlling numerous biological processes, including translation, splicing, nuclear export, and decay of target RNA decay control. The involvement of three types of proteins in m6A methylation has been documented. The first is m6A methyltransferase, which promotes this modification in RNA coded by the “Writer” gene. While METTL3, METTL14, and WTAP were documented earlier, new ones like METTL16 and RBM15 are also emerging [9–11]. The second class of protein is the m6A demethylase that removes the m6A methylation group in RNA. Coded by “Erasers,” examples of these genes include FTO and ALKBH5 [12, 13].

The third type binds with the m6A methylation site in RNA to impact a slew of functions. Their coding genes are termed “Readers.” The gene encoding the YTH domain family proteins (YTHDFs and YTHDCs subtypes) was the earliest documented. This m6A epigenetic modification vitally controls the incidence and progression of malignancies via oncogene or tumor-suppressor gene mRNA molecules to control their expression [14–16]. Yet, the role of m6A in intracranial tumors lacks comprehensive elucidation [17, 18].

Increasing data suggest that N6-methyladenosine (m6A) RNA methylation regulators have a role in carcinogenesis and tumor growth. There is currently no report of a risk model that incorporates m6A regulatory gene mRNA expression levels to investigate AS patients' prognosis. This study comprehensively analyzed the expression profiles and prognostic value of the m6A RNA methylation regulators risk score model in AS patients through several databases. Finally, the current study systematically confirmed the predictive functions of the m6A RNA methylation regulators risk score model in AS patients.

## 2. Materials and Methods

### 2.1. Data Collection

The CGGA (http://www.cgga.org.cn) and the GTEx (http://commonfund.nih.gov/GTEx/) databases were the sources of gene expression and clinical data. This was a total of 579 AS patient data, including 148 patients with astrocytoma (A, WHO grade II), 160 patients with anaplastic astrocytoma (A.A., WHO grade III), and 271 patients with glioblastoma (GBM, WHO grade IV) from the CGGA database. The control encompassed RNA transcriptome datasets of 619 normal human brain tissue specimens from the GTEx database. Standardization of these two database gene expression levels entailed the application of log2 (*X* + 1) (*X* is the original expression level of the gene). m6A RNA methylation regulators were selected based on earlier reports and gene expression data as available in the dataset [19–21]. Ultimately, 12 such regulators were included in our scrutiny.

The article "Identification of an m6A RNA Methylation Regulator Risk Score Model for Prediction of Clinical Prognosis in Astrocytoma" was retracted in 2023. Reasons: signs of a paper mill; compromised peer review; unreliable results or conclusions.

### 2.2. Differential Expression Analysis of the Regulators

After scrutinizing differentially expressed genes (DEGs) between AS vs. control datasets, the “Limma” package of *R* software was employed to test the *p* value, and a violin chart was drawn. Significance was at *p* < 0.05. Further, m6A regulator interactions were probed by the “Corrlot” and “Spearman” packages in the *R* software. The regulator expressions were compared by one-way analysis of variance and *t*-test across different clinical AS datasets with these differences illustrated in heat maps.

### 2.3. Consensus Clustering of the Regulators

The “Consensus Cluster Plus” package in the *R* software was employed to probe clusters corresponding to distinct subgroups of the regulators assayed in this work to prove their impact in AS. Following the division of patients into (*k* = 2 − 9) clusters, the survival analysis on these *k* clusters was done to scrutinize the survival time variations between groups.

### 2.4. m6A Regulatory Factor Risk Model Construction

To probe the link between m6A-related genes and prognosis, LASSO [22] and univariate Cox regression analysis were employed in the CGGA gene expression data. The genes demonstrating a significant association with the survival (*p* < 0.05) were probed to build a risk model (RS) employing the risk model formula below:

(1) $$\begin{array}{c} \text{RS}=\overset{n}{\underset{i=1}{\sum }}\text{c}\text{oefi}\times xi \end{array}$$

(coefi is the LASSO coefficient of m6A-regulated gene *i*, and *xi* is the relative expression of the m6A-regulated gene.)

The *R* survival package was employed to scrutinize the association in the CGGA database patient set between the 5-year survival rate and the R.S., the risk model (RS). The median value of the R.S. was employed to categorize patients into high-risk and low-risk groups. The Kaplan-Meier (K.M.) plot of the survival curve was constructed at *p* < 0.05. Further, the receiver operating characteristic (ROC) curve and AUC computation entailed using the survival ROC package to probe the accuracy of the survival analysis.

### 2.5. Survival Analysis of the m6A RNA Methylation Regulator Risk Model

The utility of the R.S. in AS prognosis was probed employing univariate and multivariate Cox regression analysis using the “survival” and “forest plot” software packages. Comparison of R.S., age, gender, IDH gene status, and tumor grade of the patient set entailed univariate analysis of variance and unpaired *t*-test. The Kaplan-Meier method and the log-rank test for univariate and multivariate subsistence analysis are independent prognostic factors.

The article "Identification of an m6A RNA Methylation Regulator Risk Score Model for Prediction of Clinical Prognosis in Astrocytoma" was retracted in 2023. Reasons: signs of a paper mill; compromised peer review; unreliable results or conclusions.

### 2.6. Risk Model Verification and Biological Function Analysis

The R.S. verification encompassed AS specimen data (*n* = 331) from the TCGA dataset. The R.S. formula was applied on each sample in this verification set with categorization into high-risk and low-risk groups as outlined above. Apart from the K-M diagram and ROC curve, gene set enrichment analysis employing the GSEA software v4.03 [23] was done to scrutinize the biological processes and pathways of the m6A regulatory factors in the AS in the risk model.

## 3. Results

### 3.1. The Pattern of Regulators in AS

The expression of each m6A RNA methylation regulator scrutinized of the malignant vs. control samples is depicted as a heat map (Figure 1(a)). As illustrated, the expression levels of most of these regulators demonstrated an evident correlation with AS incidence (Figure 1(b), *p* < 0.001), while AS samples showed upregulated METTL3, METTL14, WTAP, RBM15, ZC3H13, HNRNPC, YTHDF1, and YTHDF2 levels. However, opposed to controls, a downregulation of ALKBH5 and FTO also emerged (Figures 1(a) and 1(b)). Subsequent probing of the expression correlation among the 12 m6A regulators to comprehend their interactions (Figure 1(c)). The correlation plot demonstrated a strong coexpression relationship among METTL3, METTL14, WTAP, RBM15, ZC3H13, and HNRNPC. This pattern was also shown in the STRING database (Figure 1(d)).

### 3.2. Consensus Clustering and Clinical Characteristics of the Regulators in AS

This entailed the incorporation of AS patients with complete clinical information (*n* = 553) into consensus clustering analysis. In the CGGA data set, the clustering stability increased from *k* = 2 to *k* = 9, with *k* = 3 emerging an appropriate choice concerning m6A expression (Figures 2(a)–2(c)). We named them cluster 1, cluster 2, and cluster 3. Subsequently, the clinicopathological features among groups were scored (Figure 3). Evident differences among sets in age, WHO grade of tumors, and IDH gene status emerged (*p* < 0.001). While cluster 1 was associated with IDH gene mutant, cluster 3 documented an association with advanced age (age 50 years or older) and high-grade tumors.

The median survival times of cluster 1, cluster 2, and cluster 3 emerged as 20.8 months, 18.6 months, and 15.2 months, respectively, with the 5-year survival rate documenting no significant difference as per K.M. curves (*p* = 0.403). Therefore, this indicates no association between the survival time and these sample clusters (Figure 2(d)).

The article "Identification of an m6A RNA Methylation Regulator Risk Score Model for Prediction of Clinical Prognosis in Astrocytoma" was retracted in 2023. Reasons: signs of a paper mill; compromised peer review; unreliable results or conclusions.

### 3.3. DEG Selection Related to Prognosis and Risk Model Construction

From the 10 m6A-related differential genes (DEGs), a total of seven m6A-related DEGs expressive of evidence of the association with the prognosis time arose from the univariate Cox regression analysis (*p* < 0.05). Including the METTL14, WTAP, RBM15, YTHDF1, and YTHDF2 (Figure 4), the Lasso Cox regression analysis ensued to diminish model overfitting (Figures 5(a) and 5(b)). In the end, three genes WTAP, RBM15, and YTHDF2, were chosen for the R.S. model employing the formula below:

(2) $$\begin{array}{c} \text{Risk score}=\left(0.342811596553192\times \text{expression level of RBM}15\right)+\left(0.0803735398941214\times \text{expression level of YTHDF}2\right)+\left(0.0496030674327956\times \text{expression level of WTAP}\right). \end{array}$$

### 3.4. Probing the Risk Model in the Training Set

As elucidated in the materials section, following the categorization of patients into the risk groups (high and low), clinical characteristics were then scored to probe the predictive value of the three markers mentioned above in AS prognosis (Figure 6(a)). A conspicuous difference emerged for age, WHO grade of tumors, IDH gene mutant status, and tumor type (primary or recurrence) between both groups, with the high-risk group demonstrative of conspicuously elevated expression of the m6A factors assayed as opposed to the low-risk group (Figure 6(a)). The 3-year OS of the former group was 30.3% (95% Cl 25.1%, 36.7%) while that of the low-risk group was 45.1% (95% Cl 39.4%, 51.6%). The 5-year OS rates were 19.6% (95% CI: 14.8%, 26.1%) and 35.5% (95% CI: 29.7%, 42.4%) documenting a statistically significant difference (Figure 5(c), *p* < 0.01). As outlined in the materials section, the model was probed by the ROC curve with the area under ROC for a 5-year overall survival at 0.716 (Figure 5(d)).

We subsequently probed whether the risk model could be used as a risk factor independent of other clinical features. The WHO tumor stage, IDH gene mutant status, tumor type (whether primary), and the risk score documented a significant relation with the O.S. by the univariate analysis (Figure 6(b), *p* < 0.001). Subsequent multivariate Cox regression analysis revealed that the risk score remains an independent prognostic indicator of the O.S. (Figure 6(c), *p* < 0.01, H.R. = 1 1.193).

### 3.5. Corroboration of the Risk Model

The corroboration of the model entailed the AS patients samples in the TCGA database. After categorizing patients as per the risk, an apparent difference emerged for the 5-year O.S. between the high-risk and the low-risk groups (*p* < 0.01). The former group (from the target database) was demonstrative of a lower O.S. The AUC of the ROC curve of the model based on the 5-year O.S. was 0.835 (Figure 7(b)). This correlation of the O.S. with the risk model was also demonstrated by univariate regression (Figure 7(c), *p* < 0.01). As per the multivariate regression, the risk model emerged as a possible independent predictor of prognosis in AS patients after including the clinical-pathological factors (Figure 7(c), H.R. = 1.189; 95% CI: 0.825, 1.713, *p* = 0.002). These results are similar to the training set analyses outlining the stability of the constructed risk model.

The article "Identification of an m6A RNA Methylation Regulator Risk Score Model for Prediction of Clinical Prognosis in Astrocytoma" was retracted in 2023. Reasons: signs of a paper mill; compromised peer review; unreliable results or conclusions.

### 3.6. Functional Enrichment Analysis

The biological functions and pathways associated with the factors unveiled in this work were scrutinized by GSEA in the CGGA dataset. The high-risk groups demonstrated elevated expression of the biological processes related to tumorigenesis and malignancy progression (Figure 8). These were inclusive of DNA replication (NES = 1.98, *p* < 0.001), meiotic cell cycle (NES = 2.00, *p* = 0.002), nuclear chromosome segregation (NES = 2.00, *p* < 0.001), and STAT receptor signaling pathway (NES = 1.87, *p* = 0.004).

## 4. Discussion

Experimentations and analyses of the m6A modification in malignancies are still in their infancy. Given the diversity and combination of functions, the available literature does not adequately describe regulators' depth and complexity in this pathway [24, 25]. The more nuanced aspects of functions and molecules are being unveiled by employing high-throughput sequencing and other approaches in this area of science. In terms of clinical application, the scrutiny of whether m6A-related proteins can serve in diagnosis or therapy warrants detailed elucidation.

This work demonstrated the close association of m6A RNA methylation regulator expression and the occurrence and prognosis of AS. Initial regulator expression and consensus cluster analysis probing identified three AS subgroups associated with crucial clinical factors such as IDH status, tumor grade, and age. Besides, we also constructed a risk model with three such regulators and categorized AS patient data into high-risk and low-risk categories employing the risk scores. R.S. model's efficacy in AS prognosis was demonstrated using both K-M plots and the ROC curve. Its testing corroborated this on patient data from another database (TCGA), unveiling its correctness and applicability.

The article "Identification of an m6A RNA Methylation Regulator Risk Score Model for Prediction of Clinical Prognosis in Astrocytoma" was retracted in 2023. Reasons: signs of a paper mill; compromised peer review; unreliable results or conclusions.

Current research elucidates the critical role of m6A regulatory factors in carcinogenesis. These variables exhibit distinct regulation pathways across a variety of malignancies. This study discovered the increased expression of three m6A regulatory factors in the high-risk group, namely, RBM15 and WTAP (“readers”), as well as YTHDF2 (a “writer” type).

RBM15 has the most considerable weight in the risk model with its vital involvement in AS progression emerging in this work. The functioning of the human METTL3-METTL14 complex as a 6mA (DNA adenine-N6 MTase) in vitro was unveiled earlier [26]. RBM15 impacts oncogenesis by targeting the METTL3-METTL14 complex [14].

WTAP (Wilms tumor 1 associated protein) was initially identified as a splicing factor interacting with human Wilms tumor one protein [27]. The connection between its overexpression in leukemia and poor prognosis has also been documented. Elevated WTAP augments the proliferation of AML while also inducing delayed differentiation of cells [27]. Similarly, WTAP is overexpressed in cholangiocarcinoma cells, predominantly in lymph nodes or blood vessels, conspicuously augmenting their ability to migrate and invade [28]. Further, drug resistance and the power of several malignancies to proliferate, migrate, and invade are elevated by WTAP to diminish the patient's O.S. These are inclusive of pancreatic cancer, colorectal cancer, and renal cell carcinoma, to name a few [29–31]. The high expression of WTAP in GBM and its reasonable correlation with tumor progression have also been documented [32]. Our research on AS is also on these similar lines.

As an m6A reading protein, YTHDF2 can impact the target mRNA expression by recruiting a slew of regulatory or functional systems [33]. YTHDF2 upregulation in prostate cancer tissues to augment the ability of the malignant cells to divide and invade while impacting the tumor suppressor miR-493-3p expression has been corroborated [34]. The YTHDF2 expression was documented to be 83.9% in HCC patient samples with TNM stage III (*n* = 31). Subsequent assays supported the inhibition of the tumor suppressor gene miR-145 by YTHDF2 via m6A methylation to augment malignant cell proliferation [35].

Only recently has the role of RNA m6A alteration in cancers been discovered. Tumorigenesis is influenced by a myriad of critical biological processes and signaling pathways that have recently been found. Which includes cell cycle control, regeneration of tumor stem cells, DNA damage after radiotherapy, chemotherapy, cellular immune reaction, cellular hypoxia response, miRNA/lncRNA–based aspects, IL-7, STAT5, SOCS pathway, Ca2 + -mediated p-ERK12, angiogenesis, enhancer-binding protein alpha signaling pathway, and MMP9, to name a few [36, 37]. Given that m6A is receiving the limelight in studies, our transcription analysis revealed the m6A methylation regulator expression in AS progression. The roadblocks here include the paucity of studies in this sphere that necessitates the probing of additional regulators. Further additional data sets are warranted to corroborate the model developed along with appropriate wet-lab assays.

The article "Identification of an m6A RNA Methylation Regulator Risk Score Model for Prediction of Clinical Prognosis in Astrocytoma" was retracted in 2023. Reasons: signs of a paper mill; compromised peer review; unreliable results or conclusions.

## 5. Conclusion

The m6A regulatory variables are being investigated in silico to determine their expression status, prognostic significance, and biological roles. A risk model comprising three m6A regulatory genes is being developed as part of this research. The genes identified in this model can be used as new biomarkers for the prognosis of Alzheimer's disease. In addition, the identification of novel markers may make it easier for the customized prognosis of this malignancy to be incorporated into future therapy approaches. Our findings have revealed the critical role of m6A in AS oncogenesis, potentially paving the road for a cure by targeting this m6A alteration. This research provides a theoretical foundation for further fundamental medical research on m6A and AS.

## Figures and Tables

**Figure 1:** m6A RNA methylation regulator expression in AS vs. control brain and samples. (a) Heat maps of regulator expression levels of AS and control samples from CCGA and GTEx databases. (b) Corresponding violin diagrams. (c) Spearman correlation analysis of the thirteen m6A regulators (TCGA database). (d) STRING database (https://string-db.org/) documenting regulator interactions. ^∗^*p* < 0.05, ^∗∗^*p* < 0.01, and ^∗∗∗^*p* < 0.001; N: normal sample; T: tumor sample.

**Figure 2:** AS patient clustering and their overall survival (O.S.). (a) At *k* = 3, the CGGA data were categorized into three clusters. (b) Consensus clustering cumulative distribution function (CDF) for *k* = 2–9. (c) The CDF curve for *k* = 2–9 documenting the relative changes. (d) AS patient O.S. among the three clusters: K.M. plot.

**Figure 3:** The distribution of clinicopathological features and m6A regulators' expression level between different clusters.

**Figure 4:** Screening m6A-related genes linked with AS patient prognosis. The regression analyses as outlined above facilitated genes correlated with the O.S. (95% CI or confidence intervals).

**Figure 5:** Risk score model construction and scrutiny of its prognostic impact. (a, b) The risk score (R.S.) model by the LASSO Cox regression algorithm with (b) illustrative of label arrangement in the order of the lines from top to bottom. (c) K.M. plots of the CGGA set AS patient O.S. (d) ROC curve scrutinizing the prediction efficiency of the R.S. model.

The article "Identification of an m6A RNA Methylation Regulator Risk Score Model for Prediction of Clinical Prognosis in Astrocytoma" was retracted in 2023. Reasons: signs of a paper mill; compromised peer review; unreliable results or conclusions.

**Figure 6:** (a) The heat map illustrates the regulator expression across both risk groups. Comparison of the clinicopathological features between both risk groups. ^∗∗∗^*p* < 0.001. (b) Univariate Cox regression analyses for AS patient O.S. employing the R.S. and clinicopathological factors. (c) Multivariate Cox regression analyses for AS patient O.S. employing the R.S. and clinicopathological factors.

**Figure 7:** Probing the predictive risk model in the TCGA dataset. (a) AS patients of risk groups scored for O.S. by K.M. curves. (b) 5-year O.S. prediction by receiver operating characteristic (ROC) analysis l. (c, d) Univariate and multivariate Cox regression analyses of AS patient O.S. based on the R.S. (risk score) and clinicopathological factors.

**Figure 8:** The gene set enrichment analysis (GSEA) of the high-risk group.

## Data Availability

The data employed to support and corroborate the findings of this work are available from the corresponding author upon request.
